This article has been retracted.

# Sirtuin1 Role in the Melatonin Protective Effects Against Obesity-Related Heart Injury

**DOI:** 10.3389/fphys.2020.00103

**Published:** 2020-03-11

**Authors:** Gaia Favero, Caterina Franco, Alessandra Stacchiotti, Luigi Fabrizio Rodella, Rita Rezzani

**Affiliations:** ^1^Anatomy and Physiopathology Division, Department of Clinical and Experimental Sciences, University of Brescia, Brescia, Italy; ^2^Interdipartimental University Center of Research “Adaption and Regeneration of Tissues and Organs-(ARTO)”, University of Brescia, Brescia, Italy

**Keywords:** heart, melatonin, mitochondria, obesity, sirtuin1

## Abstract

Obesity is a worldwide epidemic disease that induces important structural and functional changes to the heart and predisposes a patient to devastating cardiac complications. Sirtuin1 (SIRT1) has been found to have roles in regulating cardiac function, but whether it can help in cardioprotection is not clear. The aim of the present study was to determine whether melatonin, by modulating SIRT1 and in turn mitochondria signaling, may alleviate obesity-induced cardiac injuries. We investigated 10 lean control mice and 10 leptin-deficient obese mice (*ob/ob*) orally supplemented with melatonin for 8 weeks, as well as equal numbers of age-matched lean and *ob/ob* mice that did not receive melatonin. Hearts were evaluated using multiple parameters, including biometric values, morphology, SIRT1 activity and expression of markers of mitochondria biogenesis, oxidative stress, and inflammation. We observed that *ob/ob* mice experienced significant heart hypertrophy, infiltration by inflammatory cells, reduced SIRT1 activity, altered mitochondrial signaling and oxidative balance, and overexpression of inflammatory markers. Notably, melatonin supplementation in *ob/ob* mice reverted these obesogenic heart alterations. Melatonin prevented heart remodeling caused by obesity through SIRT1 activation, which, together with mitochondrial pathways, reduced oxidative stress and inflammation.

## Introduction

Mitochondria are a major site for the generation of reactive oxygen species, which when produced in moderation have physiological roles (Sena and Chandel, 2012). If produced in excess, as occurs during aging and many pathologies, reactive oxygen species have deleterious consequences due to the damage that they inflict (Kanaan and Harper, 2017; Kauppila et al., 2017; Reiter et al., 2018). Persistent increased production of reactive oxygen species induces mitochondrial damage that, in turn, is associated with the functional decline of tissues and organs (Cardinali and Vigo, 2017). Mitochondria constitute 30% of the cardiomyocyte volume, and cardiomyocyte function is closely associated with mitochondrial activity. Consequently, mitochondrial dysfunction has been linked to heart dysfunction and remodeling (Pei et al., 2016; Gottlieb and Thomas, 2017). Our research group recently demonstrated complex mitochondrial alterations at the cardiomyocyte level of leptin-deficient obese mice (Stacchiotti et al., 2017). Accordingly, we speculated that the ethiogenesis of heart obesity-related injury is consistent with mitochondrial dysfunction and oxidative stress, even if the pathophysiological relationship among these factors awaits further elucidation.

Natural products with anti-obesity effects, especially if they lack toxicity, could be very useful in helping to prevent the growing epidemic disease of obesity (Gómez-Hernández et al., 2016; Duong et al., 2018). Ideally, a candidate would be a multitasking molecule that simultaneously exhibits antioxidant and anti-inflammatory properties, as well as having a significant impact on mitochondria. Melatonin is an attractive candidate that not only meets but also exceeds these conditions. This indoleamine is involved in a series of biological functions, including sleep regulation, blood pressure control, preservation of mitochondrial physiology, and modulation of metabolic processes, such as insulin, leptin, and lipid secretion, and has important anti-inflammatory and antioxidant protective effects (Agabiti-Rosei et al., 2017; Reiter et al., 2018; Akbari et al., 2019; Egan Benova et al., 2019). Our studies and those of other research groups obtained very promising findings regarding a potential role of melatonin in the prevention of obesity and its complications (Agabiti-Rosei et al., 2014; Favero et al., 2015; Szewczyk-Golec et al., 2015). It has been demonstrated that melatonin activates a broad spectrum of molecular pathways, including acting through sirtuin1 (SIRT1), which is an evolutionarily conserved NAD^+^-dependent deacetylase (Ramis et al., 2015; Favero et al., 2017a). Activation of AMP-activated protein kinase (AMPK) regulates SIRT1 expression. AMPK and SIRT1 together play major roles in metabolic regulation (Cantó et al., 2009; Meng et al., 2019). SIRT1 deacetylates peroxisome proliferators-activated receptor gamma coactivator 1-alpha (PGC-1α), which is a mitochondrial member of a family of transcriptional coactivators, and thereby improves metabolic signaling and mitochondrial biogenesis, and blunts pro-inflammatory pathways (Waldman et al., 2018; Zhao et al., 2019). SIRT1 is also closely involved in the control of the biological process of oxidative stress (Fry et al., 2016; Ye et al., 2019) and regulates several important transcription factors, including nuclear erythroid factor 2-related factor2 (Nrf2), which induces the transcription of antioxidant enzymes, cytoprotective factors that protect cells against oxidative stress (Tanno et al., 2010; Chong et al., 2012; Gu et al., 2016; Ye et al., 2019). Besides the profound antioxidative and anti-inflammatory effects of SIRT1, it also exhibits cardioprotective effects, but these have not been fully elucidated. Notably, SIRT1 seems involved in the cardioprotective effects of melatonin, exerting its beneficial impacts via the reduction of oxidative stress and alleviating diabetes-induced cardiac dysfunction (Ding et al., 2018; Zhang et al., 2019).

The present study uses obese mice orally supplemented with melatonin to demonstrate that melatonin effectively prevents obesity-induced heart damage through the involvement of SIRT1 activity that in turn regulates mitochondrial signaling.

## Materials and Methods

### Animal Treatment

Forty male mice, comprising 20 *ob/ob* leptin-deficient mice (B6.V-Lepob/OlaHsd) and 20 littermate lean controls, all at 4 weeks of age, were obtained from Harlan Laboratories Srl (Udine, Italy). The animals were housed in standard plastic cages in a temperature-controlled animal facility with a 12 h/12 h light–dark cycle and with free access to standard rodent chow and water. As we previously reported (Agabiti-Rosei et al., 2014; Favero et al., 2015; Stacchiotti et al., 2017), mice were randomly divided into four groups (*n* = 10 per group): (1) lean mice (treated with 1% ethanol–melatonin vehicle); (2) lean mice treated with melatonin for 8 weeks; (3) obese mice (*ob/ob*) (treated with 1% ethanol–melatonin vehicle); and (4) obese mice treated with melatonin for 8 weeks (*ob/ob*+MEL). Synthetic melatonin was dissolved in 1% ethanol and diluted in drinking water to yield a final dose of 100mg/kg body weight/day from postnatal weeks 5 to 13. Details on melatonin supplementation and rodent diet composition have been previously reported (Sartori et al., 2009; Favero et al., 2015). All the protocols were approved by the Animal Care and Use Committee of the University of Brescia (Brescia, Italy) and by the Italian Ministry of Health and comply with the commonly accepted “3Rs” indication (Replacement, Refinement, and Reduction). Systolic and diastolic blood pressures were measured non-invasively with a tail cuff device (IITC Life Science Instruments; Woodland Hills, CA, United States). At the end of the treatment period, the animals were sacrificed by cervical dislocation. Tibia lengths of the mice were measured with a digital micrometer for the calculation of the heart hypertrophy index (Zhang et al., 2015). Furthermore, blood and heart samples were collected. In particular, hearts were isolated, weighed, washed briefly in phosphate buffered saline, and frozen or immediately fixed in 4% buffered paraformaldehyde for 24 h, before being conventionally dehydrated and embedded in paraffin wax (Rezzani et al., 2013; Favero et al., 2019). Serial sections (7 μm thick) of each heart sample were cut with a microtome and submitted to morphological and immunofluorescence evaluations.

### Natriuretic Peptides Type-B Protein Level Evaluation

Homogenized heart tissues were adequately processed for the quantitative measurement of natriuretic peptides type-B (BNP) protein level using a specific ELISA Kit (Novus Biologicals, Abingdon, United Kingdom), according to the manufacturer’s instructions. The optical density value was determined using a microplate reader set at 450 nm.

### Hematoxylin–Eosin Staining

Alternate heart paraffin sections were deparaffinized, rehydrated, and stained with hematoxylin–eosin following standard protocols. The sections were then observed with an optical light microscope (Olympus, Hamburg, Germany), and the cardiomyocyte diameter was measured by counting a minimum of 20 cells containing a central nucleus on three non-consecutive sections per animal and using an image analysis program (Image Pro Premier 9.1, Media Cybernetics, Rockville, MD, United States). Furthermore, two blinded observers randomly selected five fields of three non-consecutive myocardium sections and counted the inflammatory infiltrating cells. The blinded investigators performed the analysis, and their evaluation was assumed correct if their values were not significantly different. If there was disagreement concerning the interpretation, the case was reconsidered in order to reach a unanimous agreement.

### Sirtuin1 Protein Level and Activity Analyses

Homogenized heart tissues were prepared for the quantitative measurement of the SIRT1 protein level using a SimpleStep ELISA^®^ kit (Abcam, Cambridge, United Kingdom), according to the manufacturer’s instructions. The optical density representing the SIRT1 protein level was determined using a microplate reader set at 450 nm. Furthermore, the nuclear fraction of homogenized cardiac tissue was extracted utilizing the NE-PER Kit (Thermo Fisher Scientific, IL, United States), and SIRT1 activity was measured using a specific kit assay (Abcam, Cambridge, United Kingdom) and following the manufacturer’s instructions. Nuclear SIRT1 activity was measured at 460 nm.

### Western Blot Evaluation

Homogenized heart tissues were loaded into 10% SDS-polyacrylamide gels and subjected to electrophoresis. The separated proteins were transferred to nitrocellulose membranes and then incubated with bovine serum albumin solution for 1 h, followed by overnight incubation at 4°C with the following antibodies: rabbit monoclonal AMPK (diluted 1:1,000; Cell Signaling Technology, Leiden, Netherlands), rabbit monoclonal phosphoAMPK (pAMPK; diluted 1:500; Cell Signaling Technology, Leiden, Netherlands), mouse monoclonal β-actin antibody (diluted 1:5,000; Sigma-Aldrich, St. Louis, MO, United States), and mouse monoclonal SIRT1 (diluted 1:1,000; Abcam, Cambridge, United Kingdom). Protein detection was carried out using secondary infrared fluorescent dye conjugated antibodies absorbing at 700 nm (Rezzani et al., 2019a, b). The blots were visualized using an Odyssey Fc Imaging System (LI-COR Inc., Bioscience, Lincoln, United Kingdom).

### Nuclear Erythroid Factor 2-Related Factor2 Activity Assay

Homogenized heart tissues were adequately prepared for the quantitative measurement of Nrf2 using a specific Transcription Factor Activity Assay Kit (RayBiotech Life, Peachtree Corners, GA, United States), according to the manufacturer’s instructions. The optical density representing Nrf2 activity was measured at 450 nm.

### Lipid Peroxidation Evaluation

Lipid peroxidation in heart tissue was assessed using a thiobarbituric acid reactive substance (TBARS) assay according to the formation of malondialdehyde (MDA) during acid hydrolysis of the lipid peroxide compound, as previously reported by Kaur and Muthuraman (2016). The absorbance of the organic layer was recorded at 540 nm. The TBARS level is presented as nmol/mg protein.

### Mitochondrial Reactive Oxygen Species Indicator Analyses

Reactive oxygen species were analyzed using fluorescent probe dihydrorhodamine 123 (Invitrogen; Thermo Fisher Scientific, IL, United States) applied to frozen heart sections. The sections were mounted and observed with fluorescent microscopy (i50 Eclipse, Nikon, Hamburg, Germany) at a final magnification of 400×. Twenty random fields from a total of five non-consecutive sections per animal were analyzed, and the fluorescence staining was calculated using an image analyzer (Image Pro Premier 9.1, Media Cybernetics, Rockville, MD, United States) and expressed as arbitrary units (AU). Two blinded investigators performed the analysis, and their evaluations were assumed correct if the values were not significantly different. If there was disagreement concerning the interpretation, the case was reconsidered in order to reach a unanimous agreement.

### Serum Pro-Inflammatory Cytokines Evaluation

Serum samples were obtained by collecting total blood in serum separator tubes and allowing samples to clot for 2 h at room temperature. The samples were then centrifuged for 20min at 1,000×*g*. The supernatants obtained were subjected to analyses of the levels of tumor necrosis factor-alpha (TNF-α) and interleukin-6 (IL-6) through specific ELISA assay kits and following the respective manufacturer’s instructions (Abcam, Cambridge, United Kingdom). In detail, the optical density values for TNF-α and IL-6 were determined using a microplate reader set at 450 nm.

### Immunofluorescence Analyses

Alternate heart paraffin sections were deparaffinized, rehydrated, and then incubated with the following primary antibodies: polyclonal anti-rabbit PGC-1α (diluted 1:400; Abcam, Cambridge, United Kingdom), monoclonal anti-mouse heme oxygenase-1 (HO-1) (diluted 1:400; Abcam, Cambridge, United Kingdom), polyclonal anti-rabbit Nrf2 (diluted 1:150; Abcam, Cambridge, United Kingdom), polyclonal anti-rabbit nucleotide oligomerization domain like receptor 3 (NLRP3) inflammasome (diluted 1: 600; Novus Biologicals, Abingdon, United Kingdom), polyclonal anti-goat TNF-α (diluted 1:300; Santa Cruz Biotechnology, Santa Cruz, CA, United States), and polyclonal anti-goat IL-6 (diluted 1:200; Santa Cruz Biotechnology, Santa Cruz, CA, United States). After washing, the sections were labeled with specific Alexa Fluor conjugated secondary antibodies (diluted 1:200; Invitrogen–Thermo Fisher Scientific, IL, United States) (Rodella et al., 2010, 2012). Finally, the sections were counterstained with 4′-6-diamidino-2-phenylindole (DAPI), mounted and observed with fluorescent microscopy (i50 Eclipse, Nikon, Hamburg, Germany) at a final magnification of 400× (Favero et al., 2018). Sections without primary antibody and in the presence of isotype-matched IgG served as negative immunofluorescence controls.

Twenty random fields from a total of five non-consecutive sections per animal were analyzed, and the immunostaining for each primary antibody was calculated using an image analyzer (Image Pro Premier 9.1, Media Cybernetics, Rockville, MD, United States) and expressed in AU. Two blinded investigators performed the analysis, and their evaluations were assumed correct if the values were not significantly different. If there was disagreement concerning the interpretation, the case was reconsidered in order to reach a unanimous agreement (Favero et al., 2017b; Bonomini et al., 2018).

### Statistical Analysis

Results were expressed as the mean±standard error of the mean (SEM). Data for multiple variable comparisons were analyzed by one-way analysis of variance (ANOVA corrected Bonferroni test). *p*≤0.05 was considered significant for all statistical analysis in this study.

## Results

### Heart Biometrical and Morphological Alterations

Oral treatment with melatonin for 8 weeks was well tolerated, and all animals survived up to 13 weeks of age. This observation confirmed the absence of overt side effects of melatonin supplementation (Andersen et al., 2016).

As expected, *ob/ob* mice presented higher body weight and blood pressure values in comparison to the lean mice, both supplemented and not supplemented with melatonin. Notably, melatonin supplementation markedly reduced body weight gain and systolic and diastolic pressure levels in obese mice. Furthermore, heart weight and heart hypertrophy index were also significantly increased in obese mice compared with the lean mice, both treated and not treated with melatonin. Melatonin supplementation in obese mice significantly decreased the obesity-induced rise in heart weight and heart weight to tibia length ratio.

Natriuretic peptides type-B is produced by cardiac myocytes in response to stretching of atrial or ventricular walls, and it is strongly associated with cardiovascular injury (Almuwaqqat et al., 2019). In the present study, expression of BNP was significantly lower in the heart of *ob/ob* mice compared with lean mice both supplemented and not supplemented with melatonin, and melatonin treatment of obese mice restored the BNP level. Furthermore, *ob/ob* mice also showed a higher cardiomyocyte diameter and infiltration of inflammatory cells compared to lean mice, both supplemented and not supplemented with melatonin. Notably, melatonin significantly reduced the obesity-induced cardiomyocyte diameter and inflammatory cell infiltration.

These biometric and morphometrical data are summarized in Figure 1.

**FIGURE 1:** The table summarizes biometric and morphometrical values of all experimental groups. *p≤0.05 vs lean mice, ^#^*p*≤0.05 vs lean mice supplemented with melatonin, and ^§^*p*≤0.05 vs *ob/ob* mice. Photomicrographs show representative hematoxylin–eosin stained heart sections of lean, lean mice supplemented with melatonin, *ob/ob* mice, and *ob/ob* mice supplemented with melatonin. Scale bar: 20 μm. MEL, melatonin.

As previously reported by our research group (Favero et al., 2013, 2015; Agabiti-Rosei et al., 2014; Stacchiotti et al., 2017), lean mice treated or not with melatonin displayed similar “normal” biometric and morphological data, so in the present study, they are defined generically as “lean/control” mice.

### Heart Sirtuin1 and Peroxisome Proliferators-Activated Receptor Gamma Coactivator 1-Alpha Evaluation

The heart pAMPK/AMPK ratio in *ob/ob* mice was markedly lower compared to lean mice, but melatonin supplementation in obese mice prevented the decrease in pAMPK (Figures 2A,B). *ob/ob* mice also showed a significantly reduced heart SIRT1 protein level compared to lean mice and, remarkably, obese mice supplemented with melatonin showed a completely restored SIRT1 protein concentration in the heart (Figure 2C). The same trend was observed for nuclear SIRT1 activity, summarized in Figure 2D. These observations are confirmed by SIRT1 western blot analyses (Figure 2E).

**FIGURE 2:** Representative western blot showing expression of pAMPK and AMPK in heart **(A)** of lean, *ob/ob* mice, and *ob/ob* mice supplemented with melatonin and the AMPK/pAMPK ratio as shown by relative densitometry **(B)**. The graphs summarize heart SIRT1 protein level **(C)** and activity **(D)**. Representative wester blot showing SIRT1 expression in heart of lean, ob/ob mice and ob/ob mice supplemented with melatonin **(E)**. Immunofluorescence photomicrographs of PGC-1α expression in hearts of lean **(F)**, *ob/ob* mice **(G)**, and *ob/ob* mice supplemented with melatonin **(H)**. Scale bar: 20 μm. The graph **(I)** summarizes the PGC-1α immunomorphometrical measurement. *p≤0.05 vs lean mice and #*p*≤0.05 vs *ob/ob* mice. AMPK, AMP-activated protein kinase; MEL, melatonin; pAMPK, phosphoAMP-activated protein kinase; PGC-1α, peroxisome proliferator activated receptor gamma coactivator-1alpha; SIRT1, sirtuin1.

In the present study, we also evaluated the expression of PGC-1α observing that lean mice showed a moderate expression of PGC-1α (Figure 2F), compared to a significantly decreased expression in *ob/ob* mice (very weak cardiomyocyte expression) (Figure 2G). Interestingly, melatonin supplementation in obese mice almost completely restored PGC-1α heart expression (moderate expression) (Figure 2H). These observations are also confirmed by immunomorphometrical analyses summarized in Figure 2I.

### Heart Oxidative Stress Evaluation

In the present study, we also evaluated Nrf2, a master regulator of cellular redox homeostasis (Schmidlin et al., 2019), and HO-1, one of the key enzymes that suppresses oxidative stress and may contribute to cardioprotection (Cao et al., 2015). We observed that Nrf2 was moderately/strongly expressed in the cytoplasm of lean cardiomyocytes (Figure 3A), but shows significantly decreased expression in *ob/ob* heart, reaching only very weak/weak expression (Figure 3B). Notably, melatonin supplementation in obese mice significantly increased Nrf2 expression both in the cytoplasm and the nucleus (moderate expression) (Figure 3C). These observations are confirmed by Nrf2 immunomorphometrical analyses (Figure 3D), and the same trend was observed and confirmed for Nrf2 activity, summarized in Figure 3E. Nrf2 may translocate into the nucleus to induce production of antioxidants (Silva-Islas and Maldonado, 2018). HO-1 was weakly/moderately expressed in the cytoplasm of cardiomyocytes from lean mice (Figure 3F), and its expression decreased significantly in *ob/ob* mice, with expression almost completely abolished (Figure 3G). Notably, melatonin supplementation of *ob/ob* mice induced a significant increase in the expression of HO-1 in the heart (moderate expression) (Figure 3H). These observations are confirmed also by HO-1 immunomorphometrical analyses (Figure 3I). Furthermore, obesity significantly increased oxidative stress in the heart tissue as demonstrated by increased levels of MDA (lipoprotein peroxidation) and mitochondrial reactive oxygen species in *ob/ob* mice compared with lean hearts. Notably, melatonin supplementation in obese mice reduced significantly both indicators of oxidative stress, with values reaching levels comparable to lean mice (Figures 3J,K).

**FIGURE 3:** Immunofluorescence photomicrographs of Nrf2 **(A–C)** and HO-1 **(F–H)** expression in hearts of lean **(A,F)**, *ob/ob* mice **(B,G)**, and *ob/ob* mice supplemented with melatonin **(C,H)**. Scale bar: 20 μm. The graphs summarize Nrf2 immunomorphometrical evaluation **(D)**, Nrf2 activity **(E)**, HO-1 immunomorphometrical measurement **(I)**, heart lipid peroxidation **(J)**, and mitochondrial reactive oxygen species analysis **(K)**. *p≤0.05 vs lean mice and #*p*≤0.05 vs *ob/ob* mice. HO-1, heme oxygenase-1; MEL, melatonin; Nrf2, nuclear factor erythroid-derived 2-like 2; TBARS, thiobarbituric acid reactive substance.

### Heart Inflammation Evaluation

In the present study, we observed that the NLRP3 inflammosame, which plays an important role in the development of obesity-related cardiac dysfunction and remodeling (Sokolova et al., 2019), was either absent or only very weakly expressed in the cardiomyocytes of lean mice (Figure 4A), whereas *ob/ob* mice showed moderate expression of this pro-inflammatory marker in the cytoplasm of cardiomyocytes (Figure 4B). Interestingly, NLRP3 was significantly suppressed (absent/very weak expression) in *ob/ob* mice supplemented with melatonin (Figure 4C). These observations are confirmed by NLRP3 inflammasome immunomorphometrical analyses summarized in Figure 4D. The same pattern observed for expression of the NLRP3 inflammasome was noted for TNF-α (Figures 4E–G) and IL-6 (Figures 4I–K). TNF-α is an inflammatory cytokine commonly associated with cardiac hypertrophy (Delgado et al., 2019) and along with IL-6 is involved in obesity-related alterations (Mysliwiec et al., 2018; Yarla et al., 2018). In parallel to immunomorphometrical analyses of TNF-α (Figure 4H) and IL-6 (Figure 4L), we also evaluated the serum levels of these pro-inflammatory cytokines, observing that *ob/ob* mice showed a significant increase in both TNF-α and IL-6 levels in comparison to control mice that showed very weak serum levels. Remarkably, melatonin treatment of *ob/ob* mice showed a complete restoration of TNF-α and IL-6 levels. These observations are summarized in Figures 4M,N.

**FIGURE 4:** Immunofluorescence photomicrographs of NLRP3 inflammasome **(A–C)**, TNF-α **(E–G)**, and IL-6 **(I–K)** expression at heart level of lean **(A,E,I)**, *ob/ob* mice **(B,F,J)**, and *ob/ob* mice supplemented with melatonin **(C,G,K)**. Scale bar: 20 μm. The graphs summarize the immunomorphometrical measurement of NLRP3 **(D)**, TNF-α **(H)**, and IL-6 **(L)** and serum TNF-α **(M)** and IL-6 **(N)** levels. *p≤0.05 vs lean mice and #*p*≤0.05 vs *ob/ob* mice. IL-6, interleukin-6; MEL, melatonin; NLRP3, nucleotide oligomerization domain like receptor 3; TNF-α, tumor necrosis factor-alpha.

## Discussion

The major finding from our study is that melatonin supplementation exerts cardioprotective effects, with an ability to revert heart obesogenic remodeling and injuries. *ob/ob* mice showed, together with elevated blood pressure, a higher heart weight and cardiac hypertrophic index with respect to the control lean mice, but notably, melatonin supplementation significantly attenuated these obesity-related alterations. Our observations agree with previous studies in human and animal models in which melatonin reduced blood pressure to normal ranges (Agil et al., 2011; Prado et al., 2018). In the present study, we also observed that BNP heart expression is significantly lower in *ob/ob* mice compared to lean mice. This observation is consistent with previous studies in which low levels of BNP are associated with the impairment of both systolic and diastolic cardiac function, and reduced glucose uptake and lipid accumulation (Bartels et al., 2010; Broderick et al., 2014), due to BNP possessing natriuretic and vasodilatory properties, as well as antihypertrophic effects (Gutkowska et al., 2009). Furthermore, Miyashita et al. (2009) demonstrated a significant role of signaling by this natriuretic peptide in mitochondrial biogenesis and oxygen consumption, indicating that its involvement would be beneficial against obesity. Interestingly, we observed that melatonin supplementation markedly restored BNP values in hearts of *ob/ob* mice. Notably, our research group has previously observed, in this genetically induced obese animal model, that melatonin oral supplementation hampers cardiomyocyte mitochondria remodeling and reduces hypoxia (Stacchiotti et al., 2017). Thus, we used these previous findings as a starting point for the present study, with an aim of being better able to assess the melatonin mechanism(s) of action in counteracting obesity-related heart injury.

In the present study, we observed that the development of obesity-related cardiac hypertrophy was accompanied also by an increase in mitochondrial oxidative stress and inflammation that in turn exacerbated heart morphological remodeling. All of these alterations were significantly attenuated by melatonin supplementation. In our opinion, one of the key molecules involved in the melatonin efficacy is SIRT1. We thus expanded our focus to include SIRT1, speculating that this protein might be a plausible target against obesity-induced heart injury. Its interesting role as a metabolic regulator in obesity has been previously highlighted to the extent that obesity has been defined as a SIRT1-deficient state (Schug and Li, 2011; Wang et al., 2015). In fact, obesity, metabolic syndrome, and type 2 diabetes are associated with oxidative stress and inflammation, leading to inhibition of SIRT1 (Sebastián et al., 2012; Shao et al., 2019). In the present study, we observed a significant decrease in the pAMPK/AMPK ratio in the heart, and in turn a reduction in the SIRT1 protein level and activity in *ob/ob* mice. Interestingly, melatonin reverted these alterations, restoring pAMPK and SIRT1 values to those comparable of lean mice. Overexpression or activation of SIRT1, by several activators, has been shown to effectively alleviate metabolic and cardiovascular complications in animal models of metabolic diseases, including obesity and type 2 diabetes (Schug and Li, 2011; Weisbrod et al., 2013; Fry et al., 2016). Moreover, various studies reported a rise in activity of SIRT1 in a diversity of cells/tissues and animal models after melatonin treatment (Mayo et al., 2017; Hardeland, 2018). Among many activities of SIRT1, it may regulate cellular metabolic signaling through the acetylation and activation of the coactivator PGC-1α, which induces mitochondrial transcription factors and thereby augments both mitochondrial content and cellular metabolic oxidative capacity. A close partnership between AMPK and PGC-1α also exists in regulating energy metabolism, fatty acid oxidation, and mitochondrial biogenesis (Zhang et al., 2017). As previously reported, dysfunction of this pathway has been implicated as a contributing factor in metabolic disorders (Cantó et al., 2009; de Kreutzenberg et al., 2010; Waldman et al., 2018). In the present study, we observed a decrease in PGC-1α expression in obese cardiomyocytes that, together with the high level of mitochondrial reactive oxygen species, underlined obesogenic-induced alterations at the mitochondrial level. Guo et al. (2014) reported that melatonin efficiently protected HepG2 cells against cadmium-induced mitochondrial damage by promoting SIRT1/PGC-1α signaling, indicating that melatonin can also act on mitochondria via SIRT1 (Cardinali and Vigo, 2017). Thus, in the present study, we proposed this signaling as a potential molecular mechanism of action for melatonin in the heart as well as in the liver. We highlight the importance of mitochondrial functions not only in the genesis of obesity-induced heart alterations but also notably in the protective mechanism that melatonin offers against oxidative damage. In the present study, we observed also that Nrf2, a transcription factor modulated by PGC-1α (Lin et al., 2005), is significantly reduced in the hearts of obese mice, inducing in turn a significant reduction in HO-1 expression, together with an increase in lipid peroxidation and pro-inflammatory markers, NLRP3, TNF-α, and IL-6. Interestingly, *ob/ob* mice supplemented with melatonin showed a restoration of Nrf2 expression and activity in the heart, which correlated with an increased expression of the inducible antioxidant HO-1 and a reduction in lipid peroxidation, mitochondrial reactive oxygen species, and inflammation. These important cardioprotective effects of melatonin acting through Nrf2 were recently reported by Liu et al. (2018), who observed that a melatonin-induced suppression of oxidative stress and cell death helped to protect diastolic function in high-fat-diet induced obese mice. Furthermore, previous studies have reported that HO-1 overexpression could protect the stability of the mitochondrial membrane and reduce the abundance of mitochondrial oxidation products (Chen et al., 2016; Meng et al., 2019).

Thus, our working hypothesis is presented in Figure 5, illustrating the potential mechanisms by which melatonin restores the obesity-related heart alterations in leptin-deficient obese mice. We conclude that the SIRT1/PGC-1α/Nrf2/HO-1 pathway represents a vital target in the quest to prevent adverse obesogenic cardiac remodeling. The development of novel therapeutic/protective approaches modulating this pathway may reduce the drain of health care costs and resources resulting from the worldwide spread of this epidemic disease.

**FIGURE 5:** A schematic representation of sirtuin1 involvement in the proposal melatonin mechanisms of action (blue arrows) against obesity-related cardiac injury (red arrows). AMPK, AMP-activated protein kinase; BNP, natriuretic peptides type-B; HO-1, heme oxygenase-1; mtROS, mitochondrial reactive oxygen species; NLRP3, nucleotide oligomerization domain like receptor 3; Nrf2, nuclear factor erythroid-derived 2-like 2; pAMPK, phosphoAMP-activated protein kinase; PGC-1α, peroxisome proliferator activated receptor gamma coactivator-1alpha; SIRT1, sirtuin1; TNF-α, tumor necrosis factor-alpha.

## Data Availability Statement

The datasets generated for this study are available on request to the corresponding author.

## Ethics Statement

The animal study was reviewed and approved by Animal Care and Use Committee of the University of Brescia, Brescia, Italy and by Italian Ministry of Health.

## Author Contributions

GF, LR, and RR contributed to the conceptualization and design of the experiments. GF, CF, and AS performed the experiments and formal analysis. GF wrote the draft of the manuscript. LR and RR contributed to the reviewing and editing for the manuscript. All authors read and approved the final manuscript.

## Conflict of Interest

The authors declare that the research was conducted in the absence of any commercial or financial relationships that could be construed as a potential conflict of interest.
